This article has been retracted.

# N-myc Downstream-Regulated Gene 1 (NDRG1) Regulates Vascular Endothelial Growth Factor A (VEGFA) and Malignancies in Glioblastoma Multiforme (GBM)

**DOI:** 10.1155/2022/3233004

**Published:** 2022-06-30

**Authors:** Xufan Zhang, Qian Chen, Yuchen Li, Hongqing Chen, Qin Jiang, Qiongying Hu

**Affiliations:** ^1^Department of Nuclear Medicine, Hospital of Chengdu University of Traditional Chinese Medicine, Chengdu, 610072 Sichuan Province, China; ^2^College of Medical Technology, Chengdu University of Traditional Chinese Medicine, Chengdu, 611137 Sichuan Province, China; ^3^Department of Laboratory Medicine, Hospital of Mianyang Traditional Chinese Medicine, Mianyang, 621000 Sichuan Province, China; ^4^Department of Laboratory Medicine, Hospital of Chengdu University of Traditional Chinese Medicine, Chengdu, 610072 Sichuan Province, China

## Abstract

**Background:**

NDRG1 has been reported to exhibit relatively low expression levels in glioma tissues compared with adjacent brain tissues. Additionally, NDRG1 is reported to be a tumor suppressor with the potential to suppress the proliferation, invasion, and migration of cancer cells. However, its exact roles in GBM are still unknown.

**Methods:**

Gene Expression Profiling Interactive Analysis (GEPIA) was employed to evaluate the expression level of NDRG1 in GBM. After the introduction of NDRG1, proliferation, analyses of colony formation, migration, and invasion capacities were performed. A luciferase reporter assay was performed to detect the effect of NDRG1 on the vascular endothelial growth factor A (VEGFA) promoter.

**Results:**

In this study, data from GBM and healthy individuals were retrospectively collected by employing GBM, and VEGFA was found to be differentially expressed in GBM tissues compared with adjacent brain tissues. Furthermore, NDRG1 expression is positively correlated with VEGFA expression, but not expression of the other two VEGF isoforms, VEGFB and VEGFC. In the glioma cell lines U87MG and U118, overexpression of NDRG1 significantly upregulated VEGFA. By performing a dual-luciferase reporter assay, it was observed that overexpressed NDRG1 transcriptionally activated VEGFA. Expectedly, overexpression of NDRG1 decreased cell viability by blocking cell cycle phases at G1 phase. Additionally, overexpression of NDRG1 inhibited invasion, colony formation, and tumor formation in soft agar. Remarkably, VEGFA silencing or blockade of VEGF receptor 2 (VEGFR2) further inhibited malignant behaviors in soft agar, including proliferation, invasion, colony formation, and tumor formation.

**Conclusions:**

NDRG1-induced VEGFA exerts protective effects in GBM via the VEGFA/VEGFR2 pathway. Therefore, targeting both NDRG1 and VEGFA may represent a novel therapy for the treatment of GBM.

## 1. Introduction

GBM, formerly known as pleomorphic glioblastoma, also called glioblastoma, is the most common primary malignant brain tumor [1]. It is caused by malignant transformation of astrocytomas and is the most malignant type of astrocytoma [2]. Its incidence is approximately 3.19/100,000 per year, and the prognosis is extremely poor. Its five-year survival rate is approximately 4-5%, and the two-year survival rate in clinical trials is only 26-33%.

N-myc downstream-regulated gene 1 (NDRG1) is a tumor suppressor gene with the potential to inhibit the proliferation, invasion, and migration of tumor cells. The expression of NDRG1 is positively correlated with the survival rate of patients with GBM; thus, it is considered a tumor suppressor gene in GBM. According to a report analyzing the tumor tissue specimens of GBM patients, it has been found that the overall survival (OS) of patients with high NDRG1 expression is significantly longer than that of those with low NDRG1 expression, and the NDRG1-positive cell rate is positively correlated with prolonged survival in GBM patients [3]. Yang Y et al. studied polymorphisms of the NDRG1 gene in 1,061 participants, including 558 patients with glioma and 503 healthy individuals, and determined a relationship between polymorphisms and the risk of glioma [4]. In addition, an experiment using human glioma cell lines revealed that overexpression of NDRG1 inhibits cell proliferation and invasion in a subcutaneous tumor mouse model and suppresses tumor occurrence [5]. Based on these findings, NDRG1 has been considered to be a powerful tumor suppressor in GBM and gliomas.

At present, the therapeutic efficacy for gliomas is poor, especially GBM. The recent experimental report of VEGF- or VEGF receptor- (VEGFR-) targeted therapy combined with chemotherapy in patients with malignant gliomas demonstrates that its antitumor effect and acceptable safety have reached an unprecedented level. More specifically, bevacizumab (BV) combined with irinotecan presents a 10-fold improvement in radiological response and a significant improvement in progression-free survival (PFS) and OS in patients with recurrent GBM [6, 7]. Therefore, a major current focus of neurooncology is to further develop antiangiogenic strategies.

NDRG1 plays an important role in VEGFA-induced angiogenesis. It has been shown that NDRG1 deficiency significantly attenuates VEGFA-induced angiogenesis, and NDRG1 is closely correlated with plc*γ*1, suggesting that NDRG1-mediated plc*γ*1 activation may be a reliable therapeutic target for VEGFA-mediated vascular diseases, including cancers [8].

Based on this previous research, we hypothesized that NDRG1 could exert crucial regulatory roles in GBM. The aim of this study was to investigate the potential regulatory role of NDRG1 on malignant behaviors and the downstream VEGFA/VEGFR2 axis in GBM.

## 2. Material and Methods

### 2.1. Publicly Available Datasets and Resources

The transcription data of the NDRG1 was collected from Gene Expression Profiling Interactive Analysis (http://gepia.cancer-pku.cn/index.html) [9]. The Cancer Genome Atlas (TCGA) (https://portal.gdc.cancer.gov/) was employed to collect NDRG1 RNA-seq data and related clinical information [10].

### 2.2. RNA Extraction and Quantitative Reverse Transcription-PCR Analysis (RT-qPCR)

Total RNA was isolated using an animal tissue/cell total RNA isolation kit (Cat. No.: RP003, DocSense, Chengdu, China) according to the manufacturer's instructions. Complementary DNA (cDNA) was obtained from 0.5 *μ*g of total RNA using ReverTra Ace qPCR RT Master Mix (Toyobo) according to the manufacturer's instructions. Quantitative PCR was performed using SYBR Green qPCR Master Mix (Life Technologies, USA). Briefly, qPCR was conducted in a final volume of 20 *μ*L, including 10 *μ*L qPCR Mix, 4 *μ*L primers (3.75 *μ*mol/L and 2 *μ*L each of both forward and reverse primers), 0.5 *μ*L cDNA templates, and 5.5 *μ*L distilled water. The primers are described as follows: NDRG1 5′-CTCCTGCAAGAGTTTGATGTCC-3′ and 5′-TCATGCCGATGTCATGGTAGG-3′ and VEGFA 5′-AGGGCAGAATCATCACGAAGT-3′ and 5′-AGGGTCTCGATTGGATGGCA-3′. The running procedure is described as follows: initial denaturation at 95°C for 1 min, 40 amplification cycles of real-time fluorescence measurement and denaturation at 94°C for 30 s, annealing at 55°C for 30 s, and elongation at 72°C for 30 s.

### 2.3. Lentiviral Infection and RNA Interference (RNAi)

Lentiviral particles carrying the NDRG1 vector (Ubi-MCS-3FLAG-CBh-gcGFP-IRES-puromycin-NDRG1) were constructed by GeneChem (Shanghai, China). Harvested virus was then used to infect cells. Stable clones were selected using puromycin and confirmed using Western blot. Short-hairpin RNA (shRNA) oligonucleotides targeting VEGFA were purchased from ORIGENE (Cat. No.: TL308426V, Guangzhou, China).

### 2.4. Dual-Luciferase Reporter Assay

The promoter regions of wild-type and mutant *VEGF-A* genes were cloned into the pGL4 basic luciferase reporter vector (Thermo Fisher Scientific, MA, USA) as described previously [11]. All vectors were verified by sequencing. The cells were seeded in 6-well plate and transfected with *VEGF-A* promoter luciferase reporter gene (0.5 *μ*g). 48-hour later, cell lysates were collected, and the dual-luciferase reporter assay kit (E2920, Promega, USA) was used to analyze the firefly and *Renilla* luciferase activity. The ratio of firefly-to-*Renilla* luciferase activity was used as a standardization index for the luciferase activity of each group.

### 2.5. Cell Viability Assay

For each 96-well plate, 5 × 10^3^ cells were seeded, and the viability was determined using a Cell Counting Kit-8 assay (CCK-8; Dojindo, Kumamoto, Japan) every 24 h for 4 consecutive days. Briefly, culture medium was replaced with 100 *μ*L original medium containing 10 *μ*L CCK-8 solution, and absorbance was measured on a microplate reader (Bio-Rad) at 450 nm. Five replicates of each treatment were used, and experiments were performed in triplicate.

### 2.6. Cell Cycle Distribution

Cells were pelleted and washed by precold PBS for 3 times. 1 × 10^6^ cells were collected and fixed using 1 mL of 75% ice-cold ethyl alcohol, stored overnight at 4°C for 16 h, and washed by PBS for 2 times. 100 *μ*L RNase A and 400 *μ*L propidium iodide (PI) (Sigma-Aldrich Chemical Company, St Louis, MO, USA) were added in the dark and incubated for 30 min at room temperature. After 30 min incubation at 4°C, it was measured using the FACS LSRII flow cytometer (BD Biosciences, Franklin Lakes, NJ, USA).

### 2.7. Colony Formation Assay

5 × 10^3^ cells were plated in 6-well plates and cultured for 14 days. After that, colonies were washed three times with PBS and fixed with 4% paraformaldehyde at room temperature for 10 min. Then, fixed colonies were stained with 0.5% crystal violet for 10 min at room temperature. Cell colonies with diameters >1.5 mm were counted. The experiment was performed in triplicate.

### 2.8. Transwell Assay

The cells were suspended with 0.25% Trypsin and washed with ice-cold PBS for three times. 1 × 10^4^ cells were seeded on the top chamber of inserts containing 8 *μ*M pore polycarbonate filters (Corning Incorporated, Corning, NY, USA), precoated with Matrigel membrane (BD Biosciences, Franklin Lakes, NJ, USA). Experiments were performed in triplicate. After 48 h, the cells on the upper membrane were removed and the invaded cells were fixed with 4% paraformaldehyde at room temperature for 10 min; then, fixed cells were stained with crystal violet (Beyotime Institute of Biotechnology, Beijing, China) and counted under a microscope (magnification, ×100).

### 2.9. Western Blot Analysis

To analyze protein levels, cultured cells were lysed using SoniConvert® Tissue Cell Convertor (DocSense, Chengdu, China) according to manufacturer's instruction. Briefly, 1 × 10^6^ cells were suspended using animal tissue/cells/bacteria total protein isolation kit (Cat. No.: PP003, DocSense). Protein concentrations were quantified using the Bio-Rad Protein Assay (Bio-Rad Laboratories). Equivalent quantities of lysate protein (20 *μ*g/lane) were electrophoresed using an Any kD™ Mini-PROTEAN® TGX™ Precast Protein Gel for sodium dodecyl sulfate-polyacrylamide gel electrophoresis (SDS-PAGE) and transferred to an Immuno-Blot® PVDF Membrane (Bio-Rad Laboratories). Transferred membrane was blocked with 10% skim milk powder in Tris-buffered saline for 1 h. The blots were then incubated overnight at 4°C with primary antibodies as follows: anti-NDRG1 (Cat. No.: ab124689), anti-VEGFA (Cat. No.: ab52917), anti-Cyclin D1 (Cat. No.: ab16663), anti-Cyclin E1 (Cat. No.: ab33911), anti-PCNA (Cat. No.: ab29), and anti-Ki67 (Cat. No.: 15580) at dilution of 1 : 1000. Then, membrane was incubated with anti-rabbit immunoglobulin IgG peroxidase-labeled secondary antibody at dilution of 1 : 2000. All antibodies were bought from Abcam. Immune complexes were visualized using enhanced chemiluminescence plus Western blotting detection reagents (GE Healthcare Life Sciences).

### 2.10. Statistical Analysis

All experimental results are expressed as the mean ± standard error of the mean (SEM). For experiments involving only two groups, the data were analyzed using a *t* test. Multiple comparisons were assessed using one-way analysis of variance (ANOVA) followed by Dunnett's multiple comparison test. Statistical analyses were performed using GraphPad Prism 8 (GraphPad Software, Inc.). Statistical significance was defined as *P* < 0.05.

## 3. Results

### 3.1. Expression of NDRG1 Is Significantly Correlated with VEGFA in GBM Tissues

By employing Gene Expression Profiling Interactive Analysis (GEPIA) (http://gepia.cancer-pku.cn/), we found that in GBM tissues (163 tumor tissues and 207 adjacent tissues), transcription of NDRG1 is positively correlated with VEGFA, but not VEGFB or VEGFC, which are two main isotypes of VEGF (Figure 1(a)). To understand the expression pattern of NDRG1 and VEGFA in GBM tumor, we further employed GEPIA and found that VEGFA is significantly upregulated in tumor tissues, but not NDRG1 (Figure 1(b)). As for overall survival (OS), patients in the NDRG1-low group and VEGFA-low group had a significantly better prognosis (Figure 1(c)). NDRG1 is realized as a tumor suppressor gene in GBM [R1] and contributes to better prognosis in patients, which is controversial to these results.

### 3.2. NDRG1 Transcriptionally Activates VEGFA in GBM Cell Lines

To confirm the correlation of NDRG1 with VEGFA in GBM cell lines, the expression levels of NDRG1 and VEGFA were measured in glioma cell lines Tx3868, Tx3095, U87MG, and U118. As it is illustrated in Figures 2(a) and 2(b), in U87MG and U118 cells, both NDRG1 and VEGFA presented a relative lower mRNA and protein levels. U87MG and U118 were picked for further analysis of NDRG1's role due to their relative low level of NDRG1. By performing western blot, efficient introduction of NDRG1 in both U87MG and U118 was confirmed (Figure 2(c)). Furthermore, the luciferase activity of the VEGFA reporter was activated in NDRG1-overexpressed U87MG and U118 cells (Figure 2(d)).

### 3.3. Overexpression of NDRG1 Inhibits Malignancies of GBM Cells

NDRG1 is considered as a tumor suppressor gene, including in gliomas and glioblastomas [5, 12]. Controversially, VEGFA is acting promoting roles in various kinds of tumors [13], which promotes us to further confirm whether overexpressed NDRG1 promotes malignancies in GBM. By evaluating the effects of NDRG1 on cell viability in U87MG and U118 cells, CCK-8 assay was performed and results illustrated that overexpressed NDRG1 inhibited cell viability significantly at day 4 and 5 (*p* < 0.05) (Figure 3(a)). Expectedly, overexpressed NDRG1 blocked cell cycle progression at G_1_/G_0_ phase significantly (*p* < 0.05) (Figure 3(b)). Furthermore, by detecting cell cycle-related regulator, we found that overexpressed NDRG1 decreased cyclin D1, cyclin E, PCNA, and ki-67 significantly (*p* < 0.05) (Figure 3(c)).

Then, we also detected other malignant behaviors, including invasion, colony formation, and tumor formation in soft agar. Expectedly, overexpression of NDRG1 significantly decreased all these behaviors (Figures 4(a)–4(c)).

### 3.4. Blockage of VEGFA/VEGFR2 Pathway Promotes Inhibitory Effects of Overexpressed NDRG1

We first confirmed efficient VEGFA knockdown after infection of LV-shVEGFA (Figure 5(a)) and then evaluate the effects of VEGFA knockdown or inhibition of VEGFR2 via adding Ki8751. By performing CCK-8 assay, it is observed that in NDRG1-overepressed cells, VEGFA knockdown or addition of Ki8751 significantly inhibited cell viability (Figure 5(b)). In vector-transfected cells, VEGFA knockdown or addition of Ki8751 slightly affected cell viability, potentially due to low endogenous VEGFA level (Figure 5(b)). Surprisingly, no obvious difference on cell cycle phases was observed after VEGFA knockdown of VEGFR2 inhibition in U87MG and U118 cells without NDRG1 overexpression, possibly due to low endogenous level of VEGFA (data not shown).

We then also detected the effects of VEGFA knockdown or addition of Ki8751 on invasion, colony formation, and tumor formation. Consistent with previous finding, inhibition of VEGFA/VEGFAR2 pathway further decreased all these behaviors (Figures 6(a)–6(c)).

## 4. Discussion

The presented results indicate that expression of NDRG1 exerts suppressive roles in GBM, including U87MG and U118 cells. Overexpression of NDRG1 transcriptionally activates VEGFA, but not VEGFB or VEGFC. Although overexpressed NDRG1 inhibited malignant behavior of GBM, including cell proliferation, colony formation, migration, and invasion, blockage of VEGFR2 inhibited all these behaviors even further, indicating that NDRG1-induced VEGFA may contribute to promoting angiogenesis and malignant behaviors in a VEGFA/VEFAR2 axis-dependent manner. Accordingly, we hypothesize that NDRG1 contributes to suppressing malignant behaviors in GBM. Moreover, blockade of the VEGFA/VEGFR2 axis may be a promising strategy after stimulation with NDRG1.

According to the literature, the membrane bound by the NDRG1 protein is close to the adhesion junction [14]. In cancers, the *NDRG1* gene is considered to be involved in inhibiting metastasis, which is negatively correlated with the migration of metastatic cancer cells [15–17]. Therefore, NDRG1 reduces metastatic potential by forming adhesion boundaries, increasing cell–cell adhesion, and inhibiting migration and invasion. The expression of EMT-related proteins, including vimentin, N-cadherin, and E-cadherin, as invasive markers is significantly increased in glioma cells and surgically resected specimens [18]. By analyzing migration and invasion capacities, we found that NDRG1 overexpression significantly decreased all these capacities. As a limitation, we failed to detect the expression level of EMT-related proteins.

The regulation of NDRG1 is highly complex under hypoxia, and its cellular function is still controversial. It has been demonstrated that reducing NDRG1 expression in GSCs can inhibit self-renewal, promote differentiation, and significantly inhibit tumor occurrence. In contrast, overexpression of NDRG1 in GSCs can induce PN-to-MES transition and improve the highly malignant phenotype [19]. In this study, overexpressed NDRG1 inhibited malignant behaviors, including proliferation, colony formation, tumor formation, migration, and invasion. These effects were further promoted by the addition of the VEGFR2 inhibitor Ki8751, which is similar to the effects of VEGFA knockdown. Overexpression of VEGFA is a critical regulator of EMT activation. NDRG1-induced VEGFA may promote migration and invasion; however, overexpression of NDRG1 obviously decreased migration and invasion, which is controversial regarding the effect of VEGFA on EMT. These results indicated that NDRG1 exerts regulatory roles in a VEGFA-independent manner, which is worth investigating in further studies.

Some studies have pointed out that the expression and function of NDRG1 are affected by conventional GBM treatment; thus, NDRG1 may be a promising target for GBM treatment if methods that can reduce these effects are developed in the future.

In humans, the VEGF family consists of several members: VEGF-A, VEGF-B, VEGF-C, VEGF-D, VEGF-E (viral VEGF), VEGF-F (snake venom VEGF), and placental growth factor (PlGF). Recently, endocrine gland-derived vascular endothelial growth factor (e.g., VEGF) has been added to this family. These factors show a different affinity for VEGFR subtypes. VEGF-A can activate VEGFR-1 and VEGFR-2, while VEGF-B and PlGF can only bind to VEGFR-1. Moreover, VEGF-C and VEGF-D can only bind to VEGFR-3. In this study, we revealed that NDRG1 positively correlated with the expression of VEGFA but not VEGFB or VEGFC. Overexpressed NDRG1 binds to the VEGFA promoter region and exerts transcriptional activating ability. This finding indicates its specific roles in regulating VEGFA. We hypothesized that overexpressed NDRG1 may promote angiogenesis by transcriptionally activating VEGFA. As a limitation, the expression level of VEGFA-related downstream targets involved in regulating migration and invasion should be detected in further investigation.

## 5. Conclusion

Our study demonstrates that NDRG1 exerts tumor-suppressing roles in GBM. It was also found that overexpression of NDRG1 transcriptionally activates VEGFA, which is a positive regulator of migration and invasion capacities in GBM. Stimulation of NDRG1 suppressed malignant behaviors, which was further suppressed by inhibiting VEGFA/VEGFR2 signaling. All these results provide a novel strategy for GBM therapy by stimulating NDRG1 and inhibiting VEGFA simultaneously.

## Figures and Tables

**Figure 1:** Comparison and correlation of NDRG1 with VEGFA, B, and C in GBM tissues. (a) The correlation between NDRG1 and VEGFA, B, and C were compared in GBM tissues. (b) NDRG1 and VEGFA mRNA expressions obtained from the Gene Expression Profiling Interactive Analysis database in GBM tissues (tumor *n* = 163 and adjacent tissues *n* = 207). (c) The prognostic value of NDRG1 and VEGFA in GBM tissues were obtained from GEPIA.

**Figure 2:** Detection of NDRG1 and VEGFA in glioma cell lines. (a) The mRNA levels of NDRG1 and VEGFA in Tx3868, Tx3095, U87MG, and U118 were detected by performing RT-qPCR. (b) Western blot was performed to detect NDRG1 and VEGFA protein in Tx3868, Tx3095, U87MG, and U118 cells. (c) After overexpression of NDRG1 in U87MG or U118 cells, efficient introduction of NDRG1 was detected by western blot. ^∗^*P* < 0.05 vs. vector group.

**Figure 3:** The effects of NDRG1 on cell proliferation. (a) NDRG1-overexpressed and vector-transfected cells were detected by performing CCK-8 assay from day 1 to 5. ^∗^*P* < 0.05 vs. vector group. (b) Cell cycle phases were detected by performing PI staining followed by flow cytometry. ^∗^*P* < 0.05 vs. vector group. (c) Cell proliferation-related proteins including cyclin D1, cyclin E, PCNA, and ki-67 were detected by performing western blot. ^∗^*P* < 0.05 vs. vector group.

**Figure 4:** The effects of NDRG1 on malignant behaviors. The effects of overexpressed NDRG1 on invasion (a), colony formation (b), and tumor formation on soft agar (c) were measured. ^∗^*P* < 0.05 vs. vector group.

**Figure 5:** Inhibition of VEGFA/VEGFR2 pathway promotes the inhibitory effects of overexpressed NDRG1 on cell proliferation. (a) Efficient knockdown of VEGFA by LV-shVEGFA was confirmed by western blot. ^∗^*P* < 0.05 vs. vector group. (b) Cell viability from day 1 to 5 was performed after VEFGA knockdown or inhibition by adding Ki8751. ^∗^*P* < 0.05 vs. vector group; ^#^*P* < 0.05, vector/shVEGFA group.

**Figure 6:** Inhibition of VEGFA/VEGFR2 pathway promotes the inhibitory effects of overexpressed NDRG1 on malignant behaviors. After VEGFA knockdown or inhibition of VEGFR2, malignant behaviors, including invasion (a), colony formation (b), and tumor formation in soft agar (c), were performed. ^∗^*P* < 0.05 vs. vector group; ^#^*P* < 0.05, vector/shVEGFA group.

## Data Availability

All data generated or analyzed during this study are included in this published article.
